# Isolates of Liao Ning Virus from Wild-Caught Mosquitoes in the Xinjiang Province of China in 2005

**DOI:** 10.1371/journal.pone.0037732

**Published:** 2012-05-23

**Authors:** Xinjun Lv, Fauziah Mohd Jaafar, Xiaohong Sun, Mourad Belhouchet, Shihong Fu, Song Zhang, Su-xiang Tong, Zhi Lv, Peter P. C. Mertens, Guodong Liang, Houssam Attoui

**Affiliations:** 1 State Key Laboratory for Infectious Disease Prevention and Control, Institute for Viral Disease Control and Prevention, Chinese Center for Disease Control and Prevention, Beijing, People's Republic of China; 2 Department of Vector-borne Viral Diseases, Institute for Animal Health, Pirbright, Woking, Surrey, United Kingdom; 3 Xinjiang Center for Disease Control and Prevention, Xinjiang, People's Republic of China; University of Minnesota, United States of America

## Abstract

Liao ning virus (LNV) is related to Banna virus, a known human-pathogen present in south-east Asia. Both viruses belong to the genus *Seadornavirus*, family *Reoviridae*. LNV causes lethal haemorrhage in experimentally infected mice. Twenty seven isolates of LNV were made from mosquitoes collected in different locations within the Xinjiang province of north-western China during 2005. These mosquitoes were caught in the accommodation of human patients with febrile manifestations, or in animal barns where sheep represent the main livestock species. The regions where LNV was isolated are affected by seasonal encephalitis, but are free of Japanese encephalitis (JE). Genome segment 10 (Seg-10) (encoding cell-attachment and serotype-determining protein VP10) and Seg-12 (encoding non-structural protein VP12) were sequenced for multiple LNV isolates. Phylogenetic analyses showed a less homogenous Seg-10 gene pool, as compared to segment 12. However, all of these isolates appear to belong to LNV type-1. These data suggest a relatively recent introduction of LNV into Xinjiang province, with substitution rates for LNV Seg-10 and Seg-12, respectively, of 2.29×10^−4^ and 1.57×10^−4^ substitutions/nt/year. These substitution rates are similar to those estimated for other dsRNA viruses. Our data indicate that the history of LNV is characterized by a lack of demographic fluctuations. However, a decline in the LNV population in the late 1980s - early 1990s, was indicated by data for both Seg-10 and Seg-12. Data also suggest a beginning of an expansion in the late 1990s as inferred from Seg-12 skyline plot.

## Introduction

The genus *Seadornavirus* encompasses mosquito-borne 12 segmented dsRNA viruses that have been isolated in South-east Asia. The genus is classified within family *Reoviridae*, subfamily *Sedoreovirinae* [1], and contains 3 recognised species, *Banna virus* (BAV), *Kadipiro virus* (KDV) and *Liao ning virus* (LNV) [2]. Seadornaviruses are transmitted by *Anopheles*, *Culex* and *Aedes* mosquitoes. *Banna virus*, which is the type species, has been isolated from mosquitoes in Indonesia (particularly in Java) [3], Vietnam [4] and China [5]. Structural analysis of outer-capsid proteins of BAV showed an ancestral relationship to the rotaviruses, which are non-vectored enteric dsRNA viruses also belonging to the family *Reoviridae* [6].

*Banna virus* was first isolated from cerebrospinal fluids (CSF) (2 isolates) and sera (25 isolates) of patients with encephalitis in the Yunnan province (Xishuang Banna prefecture) of southern China in 1987. It was also isolated in 1992 from patients with fever and flu-like manifestation [7] in the Xinjiang province. Numerous further isolates were obtained from human patients suffering from encephalitis [5], [8], [9]. BAV was also isolated from rodents, cattle and pigs, and from sera and CSF of humans with encephalitis and febrile illness in several other provinces of China (Beijing, Gansu, Hainan, Henan, Shanshi) and is therefore implicated as pathogenic in humans [5], [7], [10]. In contrast Kadipiro virus has only been isolated from mosquitoes [3].

Banna virus and Kadipiro virus replicate in both insect cells and in mice, although their replication in mammalian cells is restricted to BSR cells [11], [12], [13]. Liao ning virus, replicates in insect cells, in a wide range of primary and transformed mammalian cells, and in mice, causing lethal haemorrhages after two successive injections [14]. This paper describes a survey of arboviruses in North-east China, which was intended to identify emerging or re-merging viruses circulating in the region, including flaviviruses (such as Japanese encephalitis virus (JEV)), alphaviruses and Banna virus. Although JEV was not isolated during these surveys, LNV was isolated from 27 pools of mosquitoes (containing a total 3276 insects). We describe sequence analyses and phylogenetic comparisons of genome segments 10 and 12 (Seg-10 and Seg-12) from these isolates. Segment 10 encodes the cell attachment outer capsid protein of LNV and defines serotype [14]. Segment 12 of LNV encodes a non-structural protein of unknown function. Previously, sequences of segment 12 obtained from viremic animals were found to be highly diverse [14].

## Results

### Virus isolation and identification by PCR

Viruses were isolated from 27 pools of mosquitoes caught during July-August 2005 in the Kashi Prefecture of Xinjiang Province in North-west China (table 1). The viruses were all grown in *Ades albopictus* C6/36 cells, which became fusiform and detached from the culture surface. RNA preparations extracted from the infected cell-cultures were analysed by 1% agarose gel electrophoresis, in each case generating a migration pattern identical to that of the prototype isolate of LNV-1 (LNV-NE9712) (data not shown).

**Table 1:** LNV isolates made from wild-caught *Culex* mosquitoes collected between July and August 2005.

Isolate code	Virus isolate	Mosquito	Places collected	Date of collection (night of/month/year)	Number of mosquitoes per pool
J1	0507JS1	*Culex* species	Human accommodation, Qi Village, Jiashi county	8–9/07/2005	82
J2	0507JS2	*Culex* species	Human accommodation, Qi Village, Jiashi county	8–9/07/2005	88
J4	0507JS4	*Culex* species	Stock,, Qi Village, Jiashi county	8–9/07/2005	93
J24	0507JS24	*Culex* species	Stock, Tierimu Town, Jiashi County	11–12/07/2005	100
J27	0507JS27	*Culex* species	Stock, Tierimu Town, Jiashi County	11–12/07/2005	100
J29	0507JS29	*Culex* species	Stock, Tierimu Town, Jiashi County	11–12/07/2005	100
J32	0507JS32	*Culex* species	Stock, Tierimu Town, Jiashi County	11–12/07/2005	100
J35	0507JS35	*Culex* species	Stock, Tierimu Town, Jiashi County	11–12/07/2005	100
J44	0507JS44	*Culex* species	Stock, Tierimu Town, Jiashi County	11–12/07/2005	100
J54	0507JS54	*Culex* species	Stock, Tierimu Town, Jiashi County	11–12/07/2005	100
J55	0507JS55	*Culex* species	Stock, Tierimu Town, Jiashi County	11–12/07/2005	100
J59	0507JS59	*Culex* species	Stock, Tierimu Town, Jiashi County	11–12/07/2005	100
J60	0507JS60	*Culex* species	Stock, Tierimu Town, Jiashi County	11–12/07/2005	100
B5	0507BS5	*Culex* species	Stock, Boshikeranmu village	7–8/07/2005	201
B6	0507BS6	*Culex* species	Stock, Boshikeranmu village	7–8/07/2005	200
B7	0507BS7	*Culex* species	Stock, Boshikeranmu village	7–8/07/2005	233
B8	0507BS8	*Culex* species	Stock, Boshikeranmu village	7–8/07/2005	200
B9	0507BS9	*Culex* species	Human accommodation, Boshikeranmu village	7–8/07/2005	179
B10	0507BS10	*Culex* species	Stock, Boshikeranmu village	7–8/07/2005	200
J′13	0508JS13	*Culex* species	Stock, Tierimu Town, Jiashi County	15–16/08/2005	100
J′18	0508JS18	*Culex* species	Stock, Tierimu Town, Jiashi County	15–16/08/2005	100
J′36	0508JS36	*Culex* species	Stock, Tierimu Town, Jiashi County	15–16/08/2005	100
J′37	0508JS37	*Culex* species	Stock, Tierimu Town, Jiashi County	15–16/08/2005	100
J′41	0508JS41	*Culex* species	Stock, Tierimu Town, Jiashi County	15–16/08/2005	100
J′44	0508JS44	*Culex* species	Stock, Tierimu Town, Jiashi County	15–16/08/2005	100
J′46	0508JS46	*Culex* species	Stock, Tierimu Town, Jiashi County	15–16/08/2005	100
J′49	0508JS49	*Culex* species	Stock, Tierimu Town, Jiashi County	15–16/08/2005	100

RT-PCRs, using primers designed to target Seg-10 (903 bp-long) and Seg-12 (760 bp-long) of the LNV genome, generated cDNAs of the expected sizes (845 bp for Seg-10 and 675 bp for Seg-12) from all 27 virus isolates (Figure 1). However, reactions containing generic flavivirus primers, alphavirus primers, or primers designed to amplify BAV Seg-9 (Table 2), all failed to generate PCR amplicons (positive-controls included RNA from Middleburg virus [genus *Alphavirus*], yellow fever virus 17D [genus *Flavivirus*] and Banna virus [BAV-Ch] - data not shown).

**Figure 1:** PCR amplicons from segments 10 and 12 of LNV isolates from Xinjiang province. **A:** amplicon obtained using primers LNV10s/LNV10r1 (products size 845 bp), **B:** amplicon obtained using primers LNV12S/LNV10R (products size 675 bp).the PCR products were run on 1% agarose gel in TAE buffer and subsequently stained with ethidium bromide.

**Table 2:** List of primers used in PCR amplifications.

virus	Primer designation	Position/orientation	Reference sequence accession number	Sequence	Reference
Flavivirus	PF1S	8987-9006/forward	NC_002031	TGYRTBTAYAACATGATGGG	[50]
Flavivirus	PF2R	9239-9258/reverse	NC_002031	GTGTCCCADCCDGCDGTRTC	[50]
Alphavirus	M2W	164-186/forward	L01443	YAGAGCDTTTTCGCAYSTRGCHW	[51]
Alphavirus	M2W2	288-313/forward	L01443	TGYCCNVTGMDNWSYVCNGARGAYCC	[51]
Alphavirus	cM3W	568-597/reverse	L01443	ACATDAANKGNGTNGTRTCRAANCCDAYCC	[51]
BAV	9-JKT-S	* 597-618 (A) or 591-611(B)/forward	AF052033 and AF052011	TGGGATYYHAASAWGATYAAAC	[12]
BAV	9-JKT-R	* 1059-1088 (A) or 1000-1029 (B)/reverse	AF052033 and AF052011	ACTCAGTKASTACTMYCRRGGGGTGGCTTC	[12]
LNV	LNV12s1	79-101/forward	AY317110	GGAAGAATCAATGCCGTAGCCAC	[14]
LNV	LNV12r1	584-561/reverse	AY317110	GTGACGATCTTCTCTGAACCAGTG	[14]
LNV	LNV12s2	105-128/forward	AY317110	CACTGGCTCCGGCTGTAGTAACAG	[14]
LNV	LNV12r2	539-516/reverse	AY317110	CTGTTCGGATCATCTGGAATTTGA	[14]
LNV	LNV12S	13-37/forward	AY317110	CAACTTGAACTTACTGGTGTGTTTG	This study
LNV	LNV12R	687-665/reverse	AY317110	GCCTTAGAACTTAAAGTTGTGAG	This study
LNV	LNV10S	21-46/forward	AY317108	ATGAGTAACGTGACAGAGATTCGTGC	This study
LNV	LNV10R	864-839/reverse	AY317108	GTTCCCGGACTTTCACAGCTACTTTC	This study

These include previously published primers for flaviviruses, alphaviruses, Banna virus (BAV), Liao ning virus (LNV) and primers designed in this study for Liao ning virus. *: A and B, refer to genotypes (corresponding to serotypes) A and B of BAV.

### Sequence analyses

Sequence analyses of Seg-10 and Seg-12 and comparisons to published data, showed that all 27 isolates belong to LNV-1 (represented by prototype isolate LNV-9712) [14], [15]. The sequences of Seg-10 and Seg-12 from the 27 LNV isolates were deposited in Genbank database under accession numbers HM745506- HM745532and HM745533-HM745554, respectively. The level of nt identity in Seg-12 varied from 99.0% to 100% between the 27 new LNV isolates, while the level of aa identity detected in the deduced VP12 sequences, ranged from 98% to 100%. Comparisons to Seg-12 of the earlier prototype strain of LNV-1 (LNV-9712), showed lower nt identities, ranging from 94 to 94.8%, with VP12 aa identity ranged from 99.1% to 99.93% (indicating that most of the changes were ‘silent’, involving the 3^rd^ base position of the codon). When compared to Seg-12 of the unique LNV-2 isolate (LNV-NE9731), nt identity levels ranged from 87.7% to 87.8%, with 99.8% to 99.9% aa identities in VP12 (again reflecting multiple ‘silent’, third base changes).

LNV Seg-10 encodes the cell-attachment protein VP10, which determines virus serotype [14]. The level of nt identity detected in Seg-10 between the 27 new isolates ranges from 94.3% to 100%, with 99.0% to 100%aa identity in VP10. These levels are consistent with isolates from a single serotype of LNV [14] or BAV [11]. Comparisons of Seg-10 from the 27 new isolates, with the prototype strain of LNV-1 (LNV-NE9712), identified nucleotide substitutions in a total of ninety positions within the sequenced region (nt: 21–864), 76.6% of which were 3rd position changes, 7.8% 2^nd^ position and 15.6% 1^st^ position. Overall, the prototype LNV-1 and the new isolates showed 91.9% to 93.1% nt, and 94.2% to 96.6% aa identity, which is still consistent with membership of the same virus serotype (members of the same LNV serotype show >80% amino acid identity in VP10 [14], while members of the same BAV serotype show >89% amino acid identity in VP9 [11]).

Comparisons of Seg-10 and VP10 from the new LNV isolates with the prototype strain of LNV-2 (LNV-NE9731), showed nt identity levels of only 75.1% to 75.3%, and aa levels of 79% to 80% - consistent with membership of different serotypes [14]. Analysis of base changes at the 1^st^ , 2^nd^ and 3rd codon position of the 27 isolates, showed a total of 203 substitutions relative to LNV-2 (186 of which are ‘segregating’: i.e. showing more than 2 different bases [in different isolates] for the same position). Of these changes 55.4% were at the 3^rd^ position, 19.9% at the 2^nd^ position and 24.7% at the 1^st^ position.

The Tajima D test of neutrality, implemented in MEGA4, was used to assess selection. The expected value for populations that conform to a standard neutral selection model is zero [16]. However the D values for LNV Seg-10 and Seg-12 were −2.13 and −2.55 respectively which therefore reject a ‘null hypothesis’ for neutral selection.

### Sequence diversification in LNV infected mice

Previous work [14] has shown that all three BAV, KDV and LNV were able to replicate in mice and could be detected in blood a few days after intra-peritoneal injection. A high level of sequence diversification has previously been reported to occur in LNV Seg-12/VP12, after intra-peritoneal injection of the virus into mice [14]. BAV and KDV infections were not lethal, did not result in severe clinical presentations and produced protective immunity. Re-infection was not accompanied by detectable virus replication. The situation observed after LNV injection was different. Primary infection provoked a 5 days prostration after which all tested animals recovered. However, re-infection with the same serotype or a different serotype of LNV caused a generalised haemorrhage and resulted in death of the mice.

We carried out a further study, by injecting subcutaneously LNV-1 (isolate LNV-NE9712) into 4 mice, then re-isolating the virus from mouse blood (collected 3 days post-injection) on BSR and C6/36 cells. Cell culture passage one (P1) of the re-isolated virus was used for molecular studies. Amplicons (506 bp-long) obtained by nested PCR using primers LNV12s2 and LNV12r2 (Table 2) from the infected blood sample, or from the subsequent virus isolate were sequenced. A total of 37 aa changes were detected in VP12 between different clones derived from the blood sample, with only 3 clones identical to the parental sequence. In contrast all of the clones derived from the re-isolated virus P1 in BSR or C6/36 cells were identical to the sequence of the parental virus strain, indicating that passage in cell culture had a significant selective or ‘purifying’ effect.

Twenty cDNA clones were also generated (using primers LNV10S/LNV10R) for Seg-10 of the virus re-isolated in BSR or C6/36 cells. In each case, only one codon change was identified at the same position (nucleotides 64–66: GCA→AAC), changing in alanine (A, position 82) into asparagine (N), compared to all field isolates of LNV-1.

LNV was identified by RT-PCR in the spleen of injected mice, two weeks after injection. Sequencing showed that Seg-10 and Seg-12 of the virus present in the spleen, were identical to those of the virus re-isolated from the blood collected at 3 days post-injection, indicating that the highly divergent sequences were ‘bottlenecked’. All of the blood-derived sequences have been deposited in the Genbank database under accession numbers HM756693, HM756694 and HM745468 to HM745505.

A model for the structure of LNV-1 VP10, was generated using the programme ‘MODELLER’, based on the previously published atomic structure of the homologous BAV VP9 [6] (figure 2). The model indicates that aa position 82 is located within a ‘basic’ depression at the upper/outer surface of the protein trimer. As suggested previously, this basic surface is thought to interact with an ‘acidic’ receptor-molecule on the cell-surface [6]. Most 1^st^ and 2^nd^ base variations that were detected in Seg-10 of the field isolates of LNV-1 are located between nucleotides 369 and 720, which maps to the ‘head’ of the protein monomer (aa 117 to 244), not to the ‘tail’ region where the coiled coils are located.

**Figure 2:** Theoretical model of the VP10 of LNV based on the atomic structure of the homologous VP9 of BAV. **A:** the BAV VP9 atomic structure, B: theoretical model of the VP10 of LNV. The model was constructed using the programme MODELLER. The mutation (A82→N82) found in the VP10 of the virus isolated on cell culture from the mouse blood collected at 3 days post-injection and the virus identified in the spleen 2 weeks post-injection of LNV-9712, mapped to the basic (blue colour) depression on the surface of the VP10 trimer.

### Phylogenetic and genealogy analyses

For phylogenetic reconstructions, we determined the shape-parameter alpha to be used for the gamma distance. This shape parameter measures the variability of the rates-of-change between different sites within a set of sequences. When alpha is >1, most sites will have similar rates of change, although when alpha is ≤1 most sites have very low rates, but with evolutionary hot spots with higher rates [17]. The value of the shape parameter calculated for the cloned Seg-12 sequences obtained directly from mouse blood was 0.3, while that calculated for the original mosquito isolates was to 0.5. These values indicate that most sites have very low rates of change, but there are evolutionary hot spots. Calculations of the shape parameter for aa sequences of VP12 showed that the alpha value is 0.3, again suggesting conservation with certain hotspots.

The shape parameter for both the nt and aa sequences of Seg-10 derived from the mosquito isolates was 0.3. The neighbour-joining trees (figures 3 and 4) constructed using sequences of the new field isolates, confirmed their identity as LNV-1. The LNV isolates (from Jiashi and Boshikeranmu) represented a single ‘cluster’.

**Figure 3:** Phylogenetic trees for segment 10 and VP10 of LNV isolates from Xinjiang province. **A:** Phylogenetic tree based on the nucleotide sequences. **B:** Phylogentic tree based on the amino acid sequences. Bootstrap values for 500 replications are indicated at each node. The trees were constructed using the Neighbor joining method and the Kimura 2 parameters method (nucleotides) and Poisson's correction method (amino acids). Similar trees were obtained with the P-distance algorithm. The bar represents the number of substitutions per site. Isolate designations are those reported in table 2. NE-9712 (LNV-NE9712) and NE-9731 (LNV-NE9731) are prototype strains of LNV serotypes 1 and 2, respectively. The letter B in isolates designation refers to Boshikeranmu while J refers to Jiashi county.

**Figure 4:** Phylogenetic trees for segment 12 and VP12 of LNV isolates from Xinjiang province. **A:** Phylogenetic tree based on the nucleotide sequences. **B:** Phylogentic tree based on the amino acid sequences. Bootstrap values for 500 replications are indicated at each node. The trees were constructed using the Neighbor joining method and the Kimura 2 parameters method (nucleotides) and Poisson's correction method (amino acids). Similar trees were obtained with the P-distance algorithm. The bar represents the number of substitutions per site. Isolate designations are those reported in table 2. NE-9712 (LNV-NE9712) and NE-9731 (LNV-NE9731) are prototype strains of LNV serotypes 1 and 2, respectively. The letter B in isolates designation refers to Boshikeranmu while J refers to Jiashi county.

A gene genealogy analysis of Seg-10 showed that 23 of the LNV-1 isolates (out of 27 isolated in Xinjiang) form a ‘network’ with a group of 5 identical isolates that : (J59, J′13, J27, J′46 and J′44et - figure 5A). This analysis is reflected in the tree (Figure 3), which also groups all of these isolates through a common node showing 98% bootstrap confidence. Both the tree and the genealogy analyses indicate that 4 isolates (J60, J′36 and J′41 and B7) are not directly connected to the network and do not form a second network within themselves.

**Figure 5:** Genealogy of the LNV segments 12 and 10 of the isolates from the Xinjiang province. Parsimony analysis by TCS of segments 10 (A) and 12 (B) of the LNV isolates from the Xinjiang province. Connecting lines represent a nucleotide substitution. Sequenced haplotypes (oval circles), and putative ancestral virus haplotypes (small circles) are shown. In segment 10, the network show a group of 5 isolates from Jiashi, that is directly linked to other isolates from Jiashi and Boshikeranmu. Only isolates J′36, J′41, J60 and B7 do not figure in this network. In segment 12 a larger group (including 11 isolates) is linked to all remaining isolates.

Genealogy analysis of Seg-12 also shows a network, although in this case it connects all 27 isolates (figure 5B) with a group, showing highest frequency, containing 11 isolates (B6, B7, J4, J′44, J′18, J29, J′36, J′37, J′46, J55 and J60). The deepest node for the cluster of the 27 isolates in the phylogenetic tree is supported by a bootstrap confidence level of 99% (Figure 4).

Maximum clade credibility trees (figures 6 and 7) were also generated from nucleotide sequences of Seg-10 and Seg-12, through BEAST analysis. These trees were similar to the neighbor-joining trees and clearly indicate that the prototype isolate of LNV-2 (LNV-NE9731) is distinct from all other isolates described here, and that the prototype isolate of LNV-1 (LNV-NE9712) ‘roots’ the 27 new sequences whether in segment 10 or 12.

**Figure 6:** Maximum clade credibility tree based on segment 10 of LNV-1 and LNV-2 prototype isolates and including the 27 LNV isolates obtained from mosquitoes in 2005. The axis shows the estimated dates for most recent common ancestors as years before 2005. NE-9712 (LNV-NE9712) and NE-9731 (LNV-NE9731) are prototype strains of LNV serotypes 1 and 2, respectively. Values at the nodes are those for the most recent common ancestor of segment 10.

**Figure 7:** Maximum clade credibility tree based on segment 12 of LNV-1 and LNV-2 prototype isolates and including the 27 LNV isolates obtained from mosquitoes in 2005. The axis shows the estimated dates for most recent common ancestors as years before 2005. NE-9712 (LNV-NE9712) and NE-9731 (LNV-NE9731) are prototype strains of LNV serotypes 1 and 2, respectively. Values at the nodes are those for the most recent common ancestor of segment 12.

### Estimating substitution rates and demographic history

The best fit model for datasets of both Seg-10 and Seg-12 was found to be general time reversible (GTR), with a gamma distribution (*Γ*_4_) model of site variation (GTR+*Γ*_4_). Substitution rate (expressed as substitutions/site/year) in Seg-10 was 2.29×10^−4^ (95%HPD: 1.29–3.99×10^−4^). Substitution rate in Seg-12 was 1.57×10^−4^ (95%HPD: 0.54×10^−4^–4.13×10^−4^). Based on these estimates, the mean time for the most recent common-ancestor for Seg-10 of LNV is 1553 years overall (95%HPD: 500.03–2919.37), with 501 (201.52–702.71) years for Seg-10 of LNV-1, and 271 (50.38–399.92) years for Seg-10 of the isolates made in 2005. In contrast, the most recent common-ancestor of segment 12, was 710 years (95%HPD: 357.50–1024.27 years), with 260 (95%HPD: 125.23–399.74 years), years for Seg-12 of LNV-1 and 91 years (95%HPD: 24.69–227.75 years), for Seg-12 of the isolates made in 2005.

Analyses of their demographic history, using Bayesian skyline plots for both genes, indicate that the virus maintained relatively stable population sizes over the last 1553 years. However, Seg-10 and -12, both experienced a temporary population decline during the late 1980s and early 1990s (figure 8A and 8B).

**Figure 8:** Bayesian skyline plots for segments 10 (A) and 12 (B) of LNV. The Bayesian skyline plots for both genes indicated that the virus had maintained relatively stable population sizes over the last 1553 years. However, in both segments 10 and 12, data suggested a temporary population decline during the late 1980s and early 1990s. Seg-12 data also suggest that a beginning of an expansion started in the late 1990s.

## Discussion

All known seadornaviruses are able to replicate in mice causing viraemia, although isolates of *Banna virus* and *Kadipiro virus* do not cause disease in mice [12], [14]. LNV however causes lethal haemorrhage in mice (when mice are injected at two separate occasions), although death was not attributed to an antibody facilitating-effect as previously reported [14]. Although BAV can productively infect mosquito cells, the only mammalian cells in which it has been shown to replicate are BSR cells [13]. KDV has only been grown successfully in mosquito cell lines.

Isolations of LNV from *Culex* species described in this study, and from *Aedes dorsalis* mosquitoes from a previous study [14], show that LNV has a wide vector range. The mosquito *Aedes dorsalis* exists in North America, in Europe and Asia [18], [19] in a variety of brackish and fresh water habitats. The adult feeds on mammals (including humans and domestic animals) and birds, and could therefore potentially transmit LNV to these host-species. *A. dorsalis* is a vector for Western equine encephalitis virus (genus *Alphavirus*) [20], [21] and is considered as a possible North American vector for West Nile virus (genus *Flavivirus*) [22], [23].

JEV exists in an enzootic cycle between mosquitoes and pigs and/or water birds [24]. Pig farming is not practiced in Xinjiang, where sheep are the major livestock species and a search for JEV in both the human and mosquito populations in Xinjiang province was unsuccessful. However, LNV was isolated from 27 pools of wild caught mosquitoes from Xinjinag (table 1). Twenty four of these isolates from mosquitoes were collected in animal barns although 3 isolates were obtained from human accommodation. All of these isolates were identified as LNV-1 (as indicated by the high level of aa identity in the cell-attachment protein VP10). Besides mosquito vectors, the natural host or reservoir for LNV is not clearly identified. However, like Banna virus, humans, rodents, cattle and sheep [5], [9] may represent hosts of LNV.

Sequence and phylogenetic analyses indicate that different sites in Seg-10/VP10 sequences of LNV-1 have low evolutionary rates, although there are also hot spots with higher rates. These analyses also point towards purifying selection and confirm that all of the isolates belong to a single serotype.

Diversified sequences of segment 12 that were identified in the mouse blood relate to encapsidated genomic dsRNA. Viruses that contain these diverse sequences may not be viable and may not be able to reinitiate a productive infection in susceptible/permissive cells and would therefore be bottlenecked. The stability of the genome of this arbovirus also reflects the need to replicate in both the mosquito vector and a mammalian host.

Phylogenetic trees show that LNV isolates from Boshikeranmu village and Jiashi County (approximately 50 Km apart), do not form separate clusters (at the nt or aa level) either in Seg-10 or Seg-12. Clustering within the nt tree indicates that Seg-10 of some LNV-1 isolates (J′36, J′41, J60) is ancestral to the others. ‘Gene genealogy’ analysis also indicates that Seg-10 from LNV isolates J60, J′36 and J′41 and B7, is not part of a larger Seg-10 ‘network’, or any network among themselves. In contrast all of the Seg-12 sequences were connected in a single network, indicating that the Seg-12 gene pool (in Xinjiang province) is less heterogeneous than that of Seg-10. These analyses strongly indicate that reassortment events, involving exchange of Seg-10 and Seg-12, have occurred during the evolution of these virus strains.

As seen for other arboviruses, changes in vector-host densities will also influence transmission frequency and the incidence of disease. These changes will also affect the population size of the pathogen, as it follows these fluctuations [25], [26], [27]. Genetic data analyses for demographic expansion of the LNV population suggested a lack of demographic fluctuations. However, a decline in LNV population was indicated by data for both Seg-10 and -12, during the late 1980s early 1990s. It is unclear if this could be attributed to changes in the abundance or distribution of competent vectors in Northern China. It is also noticeable from the skyline plot of Seg-12 that there is a beginning of an expansion in the late 1990s.

The original LNV isolates were obtained from *Aedes dorsalis* mosquitoes in 1997, while all isolates described here were from *Culex* species in 2005. Banna virus, the prototype of genus *Seadornavirus*, was originally isolated in Indonesia in 1981, subsequently in Southern China in 1987, then 20 years later in the Northern China. The identification of LNV during 1997 [14] may be the result of a relatively recent introduction into Northern China.

Recent analyses of *Aedes aegypti* genome [28] showed that genome segment 5 of LNV (which encodes VP5, a 476 aa long non-structural protein) was found integrated in the mosquito genome in the form of two distinct but contiguous DNA inserts (aa2-aa48: 76% identity, 86% similarity and aa314-aa470: 88% identity, 93% similarity to LNV-NE9712). This finding was confirmed in an *Aedes aegypti* cell line (A20) that was cultured in 1969 from first instar larvae of the London strain of *Ae. aegypti* (colonized in 1957 [29]). The London strain also originates from West Africa. Wild caught *Ae. aegypti* mosquitoes from Pakistan were also found positive for the inserted Seg-5 sequence (data not shown). This indicates that insertion occurred before the introduction of *Ae aegypti* into [30], [31], [32] Asia which coincides with the development of shipping industry in 18^th^ and 19^th^ century, and that LNV could have originated from Africa where the *Ae aegypti* originates from.

The haemorrhage caused by the second injection of LNV into mice was not attributed to an antibody facilitating effect [14]. LNV was identified in mouse blood at 3 days post-injection. A significant level of diversification occurred during the early stages of LNV infection in mice. However, only the parental sequence was detected in Seg-12 of the virus after re-isolation in BSR or C6/36 cells, showing a strong ‘purifying’ effect. Analyses of Seg-10 from the re-isolated virus, showed an alanine to asparagine change in the deduced aa sequence (of each clone). The change maps to the surface of VP10 that is thought to interact with cell surface receptors. This aa position is also an asparagine in the published sequence of LNV-2 [14]. Both amino acids are non-charged and the significance of this change is unclear, although this might relate to the nature of the cell receptor.

Phylogenetic analyses of 40 clones of Seg-12 from mouse blood (4 mice) identified separate clusters of cDNA clones. The nucleotide sequences of mice 1, 2, 3 or 4 formed each a cluster containing sequences from a single animal. The identification of LNV in the spleen (two weeks post-injection) with identical sequences to the virus re-isolated from mouse blood, indicates that the highly divergent sequences identified directly in the blood, had been ‘bottlenecked’.

Phylogenetic analyses, genealogy, animal and cell culture work on the field samples show that LNV Seg-12 varies less than Seg-10. This mirrors findings concerning the variability of genome segments encoding cell-attachment outer-capsid proteins, of other dsRNA arboviruses, particularly the orbiviruses [33], [34], [35]. Evolutionary rates of 4 genome segments of another dsRNA arbovirus (bluetongue virus, BTV: a *Culicoides*-borne orbivirus), were previously found to be within a similar order of magnitude and ranged from 0.5×10^−4^ to 7×10^−4^ substitutions/nt/year [36].

*Banna virus* is implicated as a cause of disease in humans [5], [7], [10]. LNV is capable of replicating in a wide range of cell types, is lethal in mice and can replicate in multiple mosquito species. The recent emergence of other arboviral diseases, linked to climate change suggests that LNV could potentially emerge as an important agent of disease in animals including livestock and/or humans.

An ELISA, based on the serotype-specific protein VP10 of the two known serotypes of LNV, has been developed and is being used for epidemiological surveys of LNV in China, particularly in Xinjiang. Real time RT-PCR systems based on Seg-10 and Seg-12 of LNV have also been developed for the same purpose. These studies include humans, domesticated and wild animals (particularly rodents, sheep, birds) and will help clarify if LNV is the causative agent of disease outbreaks in China, and help to identify potential risks that may be involved. We will also attempt to identify the epidemiological impact of LNV in neighboring Asian countries.

## Materials and Methods

### Ethics statement

No specific permits were required for the described field studies. The work was done under the general supervision of the Chinese centers for disease control and prevention. No specific permission was required for trapping of mosquitoes. The trapping locations are not protected in any way. The field studies did not involve endangered or protected species.

The ethics review committee of the Institute has reviewed and approved the proposed experimental infection of LNV in mice.

### Mosquito collection, treatment and virus isolations

Mosquitoes were collected during July–August of 2005, using light traps, in human accommodations of patients with febrile manifestations, and in animal barns where sheep represent the main livestock, in Xinjiang province of China. Collections were made in Jiashi County and in Boshikeranmu village, situated in the Kashi prefecture of Xinjiang province in the north-west of China. The village and county are both located ∼50 Km from Kashi city. The collected mosquitoes were frozen for 30 min for −20°C, then sorted on an ice plate.

Blood-fed and male mosquitoes were excluded. Eighty to two hundred mosquitoes were sorted into each collecting tube and stored in liquid nitrogen.

For virus isolation, 2 ml of minimal essential medium (MEM, HyClone), supplemented with 2% foetal bovine serum, 100 U penicillin/ml and 100 U streptomycin/ml, was added to each mosquito pool, followed by homogenisation in pre-cooled sterile plastic ‘grinding’ tubes. The ground samples were centrifuged at 12,000 g for 20 min at 4°C, and the clarified supernatant was assayed for virus by inoculation onto *Aedes albopictus* C6/36 [37] mosquito cells (obtained from the American type culture collection) and BSR [38] cells (a gift from Dr. Noel Tordo, Institut Pasteur, France ). The development of cytopathic effects was followed up daily. Viruses were propagated in *Aedes albopictus* C6/36 cells at 28°C in MEM for further agarose gel electropherotyping, PCR amplifications and sequencing. Virus isolates were checked for their relatedness to Japanese encephalitis virus, Banna virus and Liao ning virus, by RT-PCR, using the primers shown in table 2.

### Inoculation of mice with LNV

The prototype strain of LNV serotype 1 (isolate LNV-NE9712: obtained from *Aedes dorsalis* mosquitoes, in the Liaoning province in northwest China in 1997) of serotype 1 was injected subcutaneously into mice. Viremic blood was collected at 3 days post-injection, before antibodies had been produced (absence of anti-LNV IgMs or IgGs: data not shown). LNV was re-isolated from mouse blood on BSR or C6/36 cells.

### Preparation of the viral RNA, reverse transcription and PCR amplification

Viral RNA was extracted from virus-infected C6/36 cells and converted into cDNA using hexaprimers as previously described [12].

RNA was extracted from mouse blood using Trizol® as previously described [12], [39].

Viral RNA was also extracted from cell cultures (BSR and C6/36) infected by the virus from mouse blood using Trizol. RNA extracts were converted to cDNA as described above.

Specific primers were designed from sequences of genome segment 12 (Seg-12) of LNV (Table 2). These were used to amplify and sequence Seg-12 from field isolates (LNV12S/LNV12R), viremic blood and cell culture re-isolated virus (first round and nested primer pairs LNV12s1/LNV12r1 and LNV12s2/LNV12r2, respectively). Primers designed from Seg-10 were only used to amplify cDNAs from virus re-isolated in cell culture. PCR was performed using the triple-master PCR (Eppendorf). Amplified products were analysed by agarose gel electrophoresis and purified by QIAquick-PCR purification (QIAGEN) and sequenced directly. Each nucleotide position was sequenced three times.

Amplicons derived from the blood and cell culture re-isolated virus were ligated into the pGEM-T vector (Promega) and transformed into bacteria. Forty plasmid clones from mouse blood (10 from each mouse) were sequenced using M13 primers. Another 80 clones from cell cultures were also sequenced (20 clones each for Seg-12 and Seg-10 from BSR cells and another 20 clones each for Seg-12 and Seg-10 from C6/36 cells).

### Sequence analysis and phylogenetic comparisons

Nucleotide (nt) and amino acid (aa) sequence alignments were generated using ClustalX version 1.8 [40]. Phylogenetic analysis was performed using MEGA4 [41], and the Neighbour-joining method was used for phylogenetic reconstructions of trees. P-distance or Kimura-2 parameters algorithms were used for the trees constructed using nucleotide sequences, while P-distance or Poisson correction algorithms were used for aa trees.

For gamma distance calculations (Kimura-2 parameter and Poisson correction models), the shape parameter alpha was determined using the PAML package [42].

Gene genealogy analysis was carried out using the programme TCS [43]. The programme collapses identical sequences into haplotypes and calculates the frequencies of the haplotypes in the sample. These frequencies are used to estimate haplotype outgroup probabilities, which correlate with haplotype age.

The best fit model of nucleotide substitution to be used in Bayesian coalescent analyses was determined using jModelTest (v 0.1.1) [44].

Bayesian coalescent analysis based on Markov Chain Monte Carlo (MCMC) sampling [45] was implemented in BEAST (Bayesian evolutionary analysis by sampling trees) [46]. Unrooted models of phylogeny and strict molecular clock models are two extremes of a continuum [47]. Substitution rates for segments 10 and 12 of LNV were therefore calculated in BEAST using a relaxed uncorrelated lognormal clock model. As applied in BEAST, this model estimates phylogenies and divergence times in the face of uncertainty in evolutionary rates and calibration times. The most general Bayesian skyline coalescent prior [48], which allows for both constant and complex changes in population size through time, was used. Differences in sampling time between 1997 and 2005 (dates of isolations of LNV strains) are used to scale branch length estimates to obtain the expected rate of genetic change per unit time. As a measure of estimate uncertainty, the program returns the 95% highest posterior density (HPD) interval. Based on the evolutionary rate, the age of the root (or of any other node) can also be estimated under the molecular clock model. In addition, the program can produce an estimate of the demographic history of the sampled population as a Bayesian skyline plot [48]. Analyses were carried out using a chain length of 10,000,000 states with the first 10% removed as burn-in. Output log files of 4 independent BEAST runs were combined together using LogCombiner (v1.5.4). This increased the effective sample sizes, and checked whether the various runs are converging on the same distribution in the MCMC run. The program Tracer (v1.5) was used to inspect posterior distributions and estimate evolutionary parameters. Maximum credibility trees were identified using TreeAnnotator (v1.5.4) and displayed using FigTree (v1.3.1).

Models for the outer capsid protein of LNV were generated using the Programme MODELLER [49] based on the previously determined atomic structure of the homologous VP9 protein of BAV.
